# A Bmi1-miRNAs Cross-Talk Modulates Chemotherapy Response to 5-Fluorouracil in Breast Cancer Cells

**DOI:** 10.1371/journal.pone.0073268

**Published:** 2013-09-09

**Authors:** Jiang Yin, Guopei Zheng, Xiaoting Jia, Zhijie Zhang, Weijia Zhang, Ying Song, Yan Xiong, Zhimin He

**Affiliations:** 1 Cancer Research Institute and Cancer Hospital, Guangzhou Medical University, Guangzhou, Guangdong, P. R. China; 2 Department of Pharmacology, Guangzhou Medical University, Guangzhou, Guangdong, P. R. China; University of South Alabama, United States of America

## Abstract

The polycomb group transcriptional modifier Bmi1 is often upregulated in numerous cancers and is intensely involved in normal and cancer stem cells, and importantly is as a prognostic indicator for some cancers, but its role in breast cancer remains unclear. Here, we found Bmi1 overexpression in 5-Fu (5-fluorouracil)-resistant MCF-7 cells (MCF-7/5-Fu) derived from MCF-7 breast cancer cells, MDA-MB-231 and MDA-MB-453 breast cancer cells compared to MCF-7 cells, was related with 5-Fu resistance and enrichment of CD44^+^/CD24^-^ stem cell subpopulation. Bmi1 knockdown enhanced the sensitivity of breast cancer cells to 5-Fu and 5-Fu induced apoptosis via mitochondrial apoptotic pathway, and decreased the fraction of CD44^+^/CD24^-^ subpopulation. In addition, our analysis showed inverse expression pattern between Bmi1 and miR-200c and miR-203 in selected breast cancer cell lines, and miR-200c and miR-203 directly repressed Bmi1 expression in protein level confirmed by luciferase reporter assay. MiR-200c and miR-203 overexpression in breast cancer cells downregulated Bmi1 expression accompanied with reversion of resistance to 5-Fu mediated by Bmi1. Inversely, Bmi1 overexpression inhibited miR-200c expression in MCF-7 cells, but not miR-203, however ectopic wild-type p53 expression reversed Bmi1 mediated miR-200c downregulation, suggesting the repressive effect of Bmi1 on miR-200c maybe depend on p53. Thus, our study suggests a cross-talk between Bmi1 and miR-200c mediated by p53, and Bmi1 interference would improve chemotherapy efficiency in breast cancer via susceptive apoptosis induction and cancer stem cell enrichment inhibition.

## Introduction

Breast cancer is the most frequently diagnosed cancer and the leading cause of cancer death in females worldwide, accounting for 23% (1.38 million) of the total new cancer cases and 14% (458,400) of the total cancer deaths in 2008 [1]. Today, although the improvement of breast cancer treatment, there are still more than 1.3 million worldwide are diagnosed with breast cancer each year and nearly half-a-million women still die from this disease each year [2]. Current treatment strategies for breast cancer combine surgery with chemotherapy and/or radiotherapy and/or hormonal therapy and/or targeted therapy. However, it is estimated that one of two breast cancer patients will fail to respond to initial treatments or will rapidly acquire resistance to un-surgery treatments [3]. Moreover, the majority of cancer patients, even if they show an initial response to chemotherapy drugs, will develop aggressive malignancies including metastasis and relapse, which exhibit up to 90% resistance to one or more drugs [4,5]. This intensely suggests that drug resistance, whether intrinsic or acquired over time, constitutes a major hurdle to successful breast cancer treatment, leading to ultimate cancer death. The underlying mechanisms of chemo-resistance are still poorly understood, although some resistance-related molecules have been identified based on established resistant-cellular models [6,7]. Several alternative but not necessarily mutually exclusive hypotheses have been proposed to explain this treatment failure and recurrence. In particular, it has been suggested that a small subpopulation of cells within tumors, termed as “tumor-initiating cells” (TICs) or “cancer stem cells” (CSCs), may be resistant to chemotherapy and hence may reinitiate tumor growth after treatment [8]. And there is increasing evidence that TICs or CSTs mediate tumor growth and metastasis and, by virtue of their intrinsic resistance to chemotherapy and radiation therapy, may also contribute to tumor recurrence [9]. In breast cancer, the CSCs population is defined as CD44^+^CD24^-^ lineage subpopulation by surface markers. In fact, chemotherapy in vitro or in vivo leads to an increase in the number of CD44^+^CD24^-^ CSCs and CD44^+^CD24^-^ CSCs appears to be more relatively resistant to chemotherapy, which represents a potentially important mechanism of acquired drug resistance in breast cancer [10,11,12]. So full understanding on CSCs may offer promise for eliciting the mechanisms of intrinsic or acquired resistance, and may also reveal the molecular targets for revising the resistance.

In recent years, growing evidence demonstrate Bmi1 (B lymphoma mouse Moloney leukemia virus insertion region 1) plays a key role in regulating and maintaining proliferation and self-renewal for normal and cancer stem cells [13,14,15]. Bmi1 is a member of the Polycomb (PcG) family of transcriptional repressors that mediate gene silencing by regulating chromatin structure [16]. Bmi1 was first described as a proto-oncogene cooperating with c-Myc during the initiation of lymphomas [17,18]. Then, Bmi1 overexpression has been frequently observed in a series of human cancers with diverse functional roles, such as non-small cell lung cancer [19], myeloid leukemia [20] and nasopharyngeal carcinoma [21]. Bmi1 is necessary for hepatic progenitor cell expansion and liver tumor development [22] and for hedgehog pathway-driven medulloblastoma expansion [23]. In addition, Bmi1 can enhance CSCs function and tumorigenicity in pancreatic adenocarcinoma [24]. Some molecular mechanisms underlying the role of Bmi1 in cancer development or progression have been proposed, such as inhibition of the tumor suppressors p16INK4a and p19ARF (p14ARF in humans) [25], and PTEN to promote EMT (epithelial-mesenchymal transition) and malignancy [26]. However, the role of Bmi1 in breast cancer chemotherapy response or resistance remains unknown. In order to explore the mechanisms responsible for acquired drug resistance in breast cancer, we have established a 5-Fu resistant-MCF-7 cell line (MCF-7/5-Fu) with typical EMT traits derived from MCF-7 breast cancer cells in our previous study [27,28]. In the present study, will first determine the expression pattern of Bmi1 in MCF-7/5-Fu and selected primary breast cancer cell lines, then investigate the role of Bmi1 in breast cancer drug resistance and the expression regulation of Bmi1-self.

## Material and Methods

### Cell culture

The human breast cancer cell lines MCF-7, MDA-MB-231 and MDA-MB-453 and the stable 5-Fu-resistant cell line MCF-7/5-Fu were cultured in RPMI-1640 (Gibco, Carlsbad, CA, USA) containing 10% fetal bovine serum (Gibco) at 37°C in a humiditied atmosphere containing 5% CO2. To maintain the resistance phenotype, 1mg/L 5-Fu (sigma) was added to the culture media for MCF-7/5-Fu cells. The human embryonic kidney cell line (HEK-293T) was cultured in DMEM (Gibco) with 10% fetal bovine serum.

### Transfection

Bmi1 expression plasmid PMSCV-BMI1 was gifted from Dr. Musheng Zeng (Sun Yat-Sen University Cancer Center, China) and short hairpin RNAs (shRNA) for Bmi1 knockdown plasmids pcDNA6.2-GW/EmGFP-shBmi1 were purchased from novobiosci (Shanghai, China). Cells were transfected with these plasmids respectively with Lipofectamine 2000 (Invitrogen) in accordance with the manufacturer’s instructions in 24-well plate. 24h later, the cells were selected with 4µg/ml puromycin and 8µg/ml Blasticidin respectively for 2 weeks and the individual stable clones were analyzed with western blot. The miR-200c mimics and miR-203 expression vector pSilencer2.1-U6-miR-203 were transfected in the 10mm dish by Lipofectamine 2000. Cells were harvested 72h later and following experiments were performed.

### MTS assay

The Cell Titer 96® AQueous One Solution Cell Proliferation Assay kit (Promega, Madison, WI, USA) was used to determine the sensitivity of cells to 5-Fu. In brief, cells were seeded in 96-well plates at a density of 4×10^3^ cells/well (0.20ml/well) for 24 h before use. The culture medium was replaced with fresh medium containing 5-Fu with different concentrations for 72h. Then, MTS (0.02ml/well) was added. After 2 h further incubation, the absorbance at 490 nm of each well was recorded on the Biotex ELX800. Growth rate was calculated as the ratio of the absorbance of the experimental well to that of the control well. The IC50 (the concentration of drug that results in 50% of control value) was also calculated.

### Real-Time PCR for Mature miRNAs and mRNAs

miRNAs from cultured cells were isolated and purified with miRNA isolation system (Exiqon). cDNA was generated with the miScript II RT Kit (QIAGEN, Hilden, Germany) and the quantitative real-time PCR (qRT-PCR) was done by using the miScript SYBR Green PCR Kit (QIAGEN) following the manufacturer’s instructions. The miRNA sequence-specific RT-PCR primers and endogenous control RNU6 were purchased from QIAGEN. The relative quantization expression was calculated by normalizing with RNU6. Total RNA was extracted with a Trizol protocol, and cDNAs from the mRNAs were synthesized with the first-strand synthesis system (Fermentas Life Science). Real-time PCRs were carried out according to the standard protocol on ABI 7500fast with SYBR Green detection (Fermentas SYBR green supermix). GAPDH was used as an internal control and the qRT-PCR was repeated three times. The primers for Bmi1 and GAPDH were showed followed: for Bmi1, forward: 5-CCACCTGATGTGTGTGCTTTG-3 and Reverse: 5-TTCAGTAGTGGTCTGGTCTTGT-3; for GAPDH: forward: 5-ATTCCATGGCACCG-3 and reverse: 5-TTCTCCATGGTGGTGAAGACGCCA-3

### FACS Analysis

The anti-CD44 (clone G44-26) and anti-CD24 (clone ML5) antibodies used for FACS analysis were obtained from BD Bioscience. Briefly, cells were incubated with trypsin–EDTA and dissociated. Cells were pelleted by centrifugation at 500 g for 5 minutes at 4°C, resuspended in 100 µL of monoclonal mouse anti-human CD24-PE antibody and a monoclonal mouse anti-human CD44-APC antibody, and incubated for 20 minutes at 4°C. The sorting was performed following the manufacturer’s instructions. Apoptosis induced by treatment with 100mg/L 5-Fu for 12h was assayed using an AnnexinV-FITC/PI Apoptosis Detection Kit (BD Pharmingen, USA) according to standard protocol with FACS analysis.

### Subcellular fractionation

After treatment, cells were washed with PBS-EDTA, trypsined, and resuspended in mitochondrial buffer containing 10 mM KCl, 0.15 mM MgCl2, 10 mM Tris-HCl pH7.6, 0.4 mM PMSF and 10 µM cytochalasin B. The cell suspensions were incubated for 30 min and homogenized on ice at 4°C with 200 strokes each in 250 mM sucrose, using a Dounce glass homogenizer. The first centrifugation was at 800 *g* for 3 min at 4°C to yield nuclei and unbroken cells as a pellet. The supernatant was centrifuged at 6,800 *g* for 10 min at 4°C and the mitochondrial pellet was resuspended in mitochondrial buffer. The cytosolic fraction was obtained as follows: cells were resuspended in Cell Free System buffer (200mMmannitol, 68mMsucrose, 2mMMgCl2, 2 mMNaCl, 2.5 mM KH2PO4, 0.5 mM EGTA, 5 mM pyruvate, 1 mM DTT, 0.1 mM PMSF and 10 mM HEPES-NaOH pH 7.4), subjected to 5 cycles of freezing/defrosting and centrifuged (150,000 *g* for 60 min at 4°C). The supernatant was kept and then submitted to western blot assay.

### Western blot assay

Cells were collected and incubated with cell lysis buffer for 20min at 4°C. Equal amount protein was added to an SDS-PAGE GEL. After electrophoresis, protein bands were transferred to PVDF membrane, blocked overnight with Tris-buffered contained 1% Tween-20 and 5% nonfat milk at 4°C. Primary antibodies used were listed as follow, p53 (cell signaling technology 1:1000); Bmi1(cell signaling technology 1:2000); cleaved-caspase7 (cell signaling technology 1:1000); cleaved-caspase9 (cell signaling technology 1:1000); β-actin(cell signaling 1:4000); Bcl-2(Santa Cruz biotechnology 1:500); Bax (Santa Cruz biotechnology 1:500). 50 micrograms total protein were loaded and separated in 10% SDS-PAGE. Anti-mouse and anti-rabbit second antibodies were purchased from Merck (Merck KGaA, Darmstadt, Germany). The signal was detected using the chemiluminescent detection system as described by the manufacturer.

### Luciferase reporter assay

Four single strands of the wild type 3’ UTR with miR-200c and miR-203 binding sites and four single strands of the mutant type with 7 bases deleted in the miR-200c and miR-203 binding sites (as mutant control) respectively, of Bmi1 were synthesized with restriction sites for SpeI and HindIII located at both ends of the oligonucleotides for further cloning. The single strand DNA sequences were following: the wild type 3’ UTR of Bmi1 for miR-200c (Sense: 5’-*CTAGT* ATTGGTATATGACATAACAGGAAAC A G T A T TGTATGATATATTTATAAATGCTATA-3’; antisense: 5’-AGCTTATAGCATTTATAAATATATCATAC A A T A C T GTTTCCTGTTATGTCA TATACCAATA-3’) and the mutated type 3’ UTR of Bmi1 for miR-200c (Sense: 5’-*CTAGT* ATTGGTATATGACATAACAGGAAA-------GTATGATATATTTATAAATGCTATA-3’; antisense: 5’-AGCTTATAGCATTTATAAATATATCATAC-------TTTCCTGTTATGTCATATACCAATA-3’); the wild type 3’ UTR of Bmi1 for miR-203 (Sense: 5’-CTAGTGTATGGGAAAATTGTAGCTAAAC A T T T C ATTGTCCCCAGTCTGCAAAAGAAGCAA-3’; antisense: 5’-AGCTTTGCTTCTTTTGCAGACTGGGGACAAT G A A A T GTTTAGCTACAATTTTC CCATACA-3’ the mutated type 3’ UTR of Bmi1 for miR-203 (sense: 5’-CTAGTGTATGGGAAAATTGTAGCTAAA-------TTGTCCCCAGTCTGCAAAAGAAGCAA-3’; antisense: 5’-AGCTTTGCTTCTTTTGCAGACTGGGGACAA-------TTTAGCTACAATTTTCCCATAC*A*-3’). The corresponding sense and antisense strands were annealed and subsequently cloned into pMir-Report plasmid downstream of firefly luciferase reporter gene. Cells were seeded in 96 well-plates and co-transfected with pMir-Report luciferase vector, pRL-TK Renilla luciferase vector and miR-200c mimics or miR-203 expression vector. 48h later the luciferase activities were determined using a Dual-Luciferase Reporter Assay System (Promega) where the Renilla luciferase activity was used as internal control and the firefly luciferase activity was calculated as the mean ± SD after being normalized by Renilla luciferase activity.

### Co-immunoprecipitation assay

Co-immunoprecipitation assay was performed followed the manual protocol. Briefly, the cells were lysed. Total protein was obtained from MCF7 cells. The immunoprecipitations were performed overnight at 4 °C with antibodies to Bmi1 or IgG (as a control). The immunopreciptates were then incubated for 2h with protein G-agarose (Promega, USA). Products were washed with lysis buffer, and the immune complexes were resolved by SDS-PAGE. Western blot assay were subsequently performed.

### Statistical analysis

Each experiment was repeated three times. Statistical analysis was carried out using SPSS 16.0. Student’s t-test was chosen to analyze the statistical difference. Results were presented as mean±SD. P<0.05 was considered statistically significant.

## Results

### Bmi1 contributes to resistance to 5-Fu and BCSCs traits maintain in breast cancer cells

To elucidate the role of Bmi1 in breast cancer cells, we first used real-time PCR and western blot to determine Bmi1 expression in MCF-7, MCF-7/5-Fu, MDA-MB-231 and MDA-MB-453 breast cancer cells with differential sensitivity to 5-Fu. As showed in Figure 1A, there was no significant differential expression of Bmi1 in mRNA levels between selected cell lines; however, Bmi1 protein was overexpressed in MCF-7/5-Fu, MDA-MB-231 and MDA-MB-453 cells compared to MCF-7 cells. Consistently, survival-concentration curves and calculated IC50 values showed MCF-7/5-Fu, MDA-MB-231 and MDA-MB-453 cells are more resistant to 5-Fu (Figure 1B). To confirm the role of Bmi1, gain-of-function and loss-of-function approaches with Bmi1 overexpression vector and Bmi1-targeting-shRNA expression vectors were used, and 2#shRNA had the most effect and was selected for following experiments (Figure 1C). We found ectopic expression of Bmi1 enhanced MCF-7 resistant to 5-Fu, and Bmi1 knockdown with shRNA sensitized MCF-7/5-Fu, MDA-MB-231 and MDA-MB-453 cells to 5-Fu (Figure 1D). Expectedly, we observed Bmi1 enriched breast cancer stem cell CD44^+^/CD24^-^ subpopulation in MCF-7 cells. However, Bmi1 knockdown declined CD44^+^/CD24^-^ subpopulation in MCF-7/5-Fu, MDA-MB-231 and MDA-MB-453 cells lines (Figure 1E). But Bmi1 had no significant effect on cell phenotype change. These results strongly implied intense association between Bmi1 and resistance to 5-Fu and CSCs enrichment in breast cancer cells.

**Figure 1:** Bmi1 expression pattern and its role in 5-Fu resistance in breast cancer cells. (A) mRNA (up) and protein (down) expression levels of Bmi1 in selected breast cancer cells; (B) Dose-survival index curves (up) were plotted from MTS assay results from three independent experiments and IC50 values (down) for 5-Fu were calculated in selected cell lines with differentail expression of Bmi1, vs MCF-7, * p<0.05, ** p<0.01; (C) MDA-MB-231 cell line was selected for verifying the knockdown efficiancey of Bmi1 specific shRNAs; (D) Dose-survival index curves (left) were plotted from MTS assay results from three independent experiments and IC50 values (right) for 5-Fu were calculated in ectopic Bmi1 overexpressed or Bmi1 knockdown cell lines, vs control, * p<0.05; (E) FACS analysis of cell-surface marker CD44 and CD24 in cell lines to indicate the breast cancer stem cell subpopulation.

### Bmi1 repressed apoptosis induced by 5-Fu through mitochondrial apoptotic pathway in breast cancer cells

As showed above, Bmi1 can mediate breast cancer cells resistant to 5-Fu, but the molecular mechanisms remains unclear. The antiapoptotic activity was measured via V-FITC/PI Apoptosis Detection Kit using Flow Cytometry. After being treated with 100mg/L 5-Fu for 12h, despite increased apoptosis in all selected cell lines, the apoptotic rate of MCF-7 was much higher than that of ectopic Bmi1 overexpressed MCF-7 cells and apoptotic rate of cell lines with Bmi1 knockdown was much higher than that of controlled cell lines, so as the total cell death rate (Figure 2A). In regard to apoptotic mechanism, we then focused on mitochondrial apoptotic pathway whether changed by Bmi1. We found Bmi1 positively regulated Bcl2 expression and the inverse relationship between Bmi1 and Bax expression also was observed (Figure 2B). Furthermore, we found Bmi1 was inversely related with cytochrome-C release and casepase9 and caspase7 activation after 100mg/L 5-Fu treatment on selected cell lines for 24h (Figure 2C and D), suggesting Bmi1 affect the mitochondrial apoptotic pathway induced by 5-Fu in breast cancer cells.

**Figure 2:** Bmi1 affects the mitochondrial apoptotic pathway in breast cancer cells. (A) Effects of 100mg/L on selected cell lines with different Bmi1 expression level. After exposure to 100mg/L 5-Fu for 12h, cells were harvested and cell death were measured with Apoptosis Detection Kit and each figures represents three independent experiments; (B) Western blot showed the reverse relationship between Bmi1 and apoptosis related molecules Bcl2 and Bax in selected cell lines; (C) Western blot showed cytochrome-C (Cyto-C) release and Caspase 9 and Caspase 7 activation after 100mg/L 5-Fu treatment on selected cell lines; (D) Effect of Bmi1 on 5-Fu-induced caspase 9 and caspase 7 activation on selected cell lines. The relative activation of caspase 9 and caspase 7 was calculated from the average of three experiments, versus control, * p<0.05, ** p<0.01.

### MiR-200c and miR-203 directly target Bmi1 expression

Because of the important role of Bmi1 in drug resistance and comparable overexpression of Bmi1 in breast cancer cells with comparable more resistant to 5-Fu, the exploration of mechanisms responsible for Bmi1 expression seems extremely necessary. There was no differential mRNA expression in selected cell lines (Figure 1A), so we focused on miRNAs which usually bind to the 3′-untranslated region (3′UTR) of target mRNA, leading to translational repression. The bioinformatic analysis using the public database-TargetScan (http://www.targetscan.org) combined with differential expression miRNAs screen using miRNA microarray between MCF-7 and MCF-7/5-Fu cells (data not shown) suggested miR-200c and miR-203 maybe target Bmi1, because Bmi1 possessed critically conserved nucleotides indicative of a legitimate target of miR-200c and miR-203 (Figure 3A). Accordingly, miR-200c and miR-203 were significantly downregulated in MCF-7/5-Fu, MDA-MB-231 and MDA-MB-453 cell lines compared to MCF-7 cells (Figure 3B). Both 40nM miR-200c mimics and pSilencer2.1-U6-miR-203 vector significantly increased miR-200c and miR-203 expression respectively (Figure 3C). Expectedly, miR-200c and miR-203 overexpression effectively inhibited Bmi1 protein in MCF-7/5-Fu, MDA-MB-231 and MDA-MB-453 cells respectively (Figure 3D). To assess whether miR-200c or miR-203 directly regulates Bmi1 expression through target the binding site in the 3’ UTR of Bmi1 mRNA, a luciferase reporter vector with the putative Bmi1 3’ UTR target site for miR-200c or miR-203 downstream of the luciferase gene (pMir-Bmi1-Wt) and mutant version thereof with a deletion of nucleotieds in the seed region was constructed (pMir-Bmi1-Mut). HEK293T cells were co-transfected with Luciferase reporter vector, pRL-TK Renilla luciferase vector and miR-200c mimics or miR-203 expression vector or control. These results showed miR-200c and miR-203 can reduce the luciferase activity of the vector with the wild-type Bmi1 3’ UTR by 65% and 53%, but the mutant version abrogated the repressive ability of miR-200c and miR-203 respectively (Figure 3E and F). These results strongly demonstrated the specificity of miR-200c and miR-203 targeting Bmi1.

**Figure 3:** miR-200c and miR-203 target Bmi1 expression. (A) Schematic of predicted miR-200c and miR-203 sites in the human Bmi1 3′UTR broadly conserved among vertebrates; (B) miR-200c and miR-203 expression status in selected cell lines, verse MCF-7 * p<0.01; (C) miR-200c mimics and miR-203 expression vector increased miR-200c and miR-203 expression, verse control * p<0.01; (D) Inverse relationship between miR-200c and miR-203 and Bmi1 protein levels was showed; (E) and (F) Mir-200c and miR-203 suppressed the activity of the luciferase gene linked by the 3′UTR of Bmi1 respectively and a Renilla luciferase reporter for normalization. The data was obtained from three independent experiments. The mean of the results from 293T cells transfected with pMir-control and miR-200c mimics or pSlience-miR-203 were set as 1.0 respectively, * p<0.01.

### Bmi1 feedback inhibits miRNA200c through p53 modulation

In the present study, low expression of miR-200c and miR-203 contributed to overexpression of Bmi1, however, whether Bmi1 feedback inhibits miR-200c and miR-203 expression to form a stable regulatory loop remains to be studied. To address the question, we detected the expression of miR-200c and miR-203 in Bmi1 interfered breast cancer cells. We found ectopic overexpression of Bmi1 downregulated miR-200c expression in MCF-7 cells but not miR-203 and Bmi1 knockdown upregulated miR-200c but not miR-203 in MCF-7/5-Fu, MDA-MB-231 and MDA-MB-453 cells (Figure 4A). Change et al. have reported p53 could positively regulate miR-200c expression at transcriptional level [27]. Coincidently, p53 was downregulated in MCF-7/5-Fu cells compared to MCF-7 cells possessing wild-type p53 (Figure 4B). To ascertain whether p53 regulates miR-200c expression in breast cancer cells, a series of experiments were performed. As shown, ectopic expression of wild-type p53 (WTp53) with pEGFP-N1-p53 vector (Figure 4B) upregulated miR-200c expression in MCF-7 and MCF-7/5-Fu cells and effectively restored Bmi1 induced miR-200c inhibition in MCF-7 cells (Figure 4C). Moreover, ectopic expression of wild-type p53 also exactly upregulated miR-200c expression in MDA-MB-231 and MDA-MB-453 cell lines, both of which posses mutational p53 and so GFP screen under fluorescence microscope used to monitor WTp53 expression after transfection (Figure 4D and E). To verify Bmi1 regulates miR-200c expression via p53 modulation, we found ectopic expression of Bmi1 factually led to p53 protein decrease in MCF-7 cells and Bmi1 knockdown led to p53 protein accumulation in MCF-7/5-Fu cells (Figure 4F). Furthermore, coimmunoprecipitation experiment showed p53 was detected in the anti-Bmi1 immunoprecipitation complex (Figure 4G), implying Bmi1 maybe mediate p53 downregulation in wild-type p53 breast cancer cells to inhibit miR-200c expression.

**Figure 4:** Bmi1 inhibits miR-200c expression via p53 downregulation. (A) the inverse expression pattern between Bmi1 and miR-200c was showed; (B) p53 protein was downregulated in MCF-7/5-Fu cells, and pEGFP-N1-WTp53 transfection increased p53 protein in MCF-7 and MCF-7/5-Fu cells, respectively; (C) WTp53 upregulated miR-200c expression and restored Bmi1 mediated miR-200c downregulation; (D) GFP screen under fluorescence microscope to monitor ectopic WTp53 expression; (E) Ectopic expression of WTp53 upregulated miR-200c in MDA-MB-231 and MDA-MB-453 with mutational p53; (F) Bmi1 negatively regulated p53 protein expression; (G) coimmunoprecipitation showed Bmi1 interacted with p53 physically. All data was obtained from three independent experiments * p<0.05, * p<0.01.

## Discussion

Chemotherapy resistance has being the major obstacle for effective breast cancer treatment. However, the mechanisms responsible for chemotherapy resistance is far from full understand. In order to explore the mechanisms responsible for acquired drug resistance in breast cancer, in our previous study, we have established a 5-Fu resistant-MCF-7 cell line (MCF-7/5-Fu) which shows typical EMT traits derived from MCF-7 breast cancer cells [28,29]. EMT process is usually accompanied with stem cell traits, so we suppose whether Bmi1 participates in the drug resistance maintain because of its important role in normal and cancer stem cells. In the present study, MCF-7, MCF-7/5-Fu, MDA-MB-231 and MDA-MB-453 cell lines with different resistance potential to 5-Fu were employed as research model to investigate the role of Bmi1 in drug resistance in breast cancer. Here, we showed the inverse Bmi1 expression pattern and 5-Fu effect and CD44^+^/CD24^-^ breast cancer stem cell population. In addition, Bmi1 knockdown sensitized breast cancer cells to 5-Fu via enhanced mitochondrial apoptotic pathway activation with Bcl2 downregulation and Bax upregulation and subsequent cytochrome-C release and caspase 9 and caspase 7 activation after 5-Fu treatment.

As for the expression regulation of Bmi1-self, we focused on miRNAs which usually elicit their regulatory effects in post-transcriptional regulation of genes by binding to the 3′-untranslated region (3′UTR) of target messenger RNA (mRNA), mainly leading to translational repression or target mRNA degradation [30]. Biologically and clinically, a large amount of literatures have reported the important role of miRNAs in chemotherapy resistance [31,32]. Specific miRNAs have altered expression in drug-resistant cancer cells. For example, miR-34a was downregulated in drug resistant prostate cancer cells and ectopic expression of miR-34a resulted in growth inhibition and sensitized cells to camptothecin [33]. Furthermore, miRNAs also modulate the EMT (Epithelial-mesenchymal transition) process and cancer stem cell program to influence the chemotherapy response to cancer treatment. Such as, Adam et al. showed miR-200 regulated EMT in bladder cancer cells and reversed resistance to EGFR inhibitor therapy [34]. Expectedly, our analysis demonstrated both miR-200c and miR-203 could directly target Bmi1 expression in breast cancer cells. MiR-200c mediated Bmi1 regulation was consistent with published reports, but miR-203 as Bmi1 regulator was identified by us for the first time [35]. Loss of miR-200c expression has been linked with cancer progression and chemotherapy resistance via EMT process and CDCs regulation [36,37]. Resent findings also strongly suggest loss of miR-200c expression contribute to drug resistance [38]. Emerging evidences suggest the implication of miR-203 expression loss in cancers, such as cancer cell proliferation, invasion and drug resistance [39,40,41], but the exact mechanism is still unclear. Here, our results showed miR-203 targeted Bmi1 to elicit its role in breast cancer drug resistance. Interestingly, we found Bmi1 inhibited miR-200c expression, but not miR-203. Chang et al have reported p53 could positively regulate miR-200c [27], and here ectopic wild-type p53 expression factually upregulated miR-200c expression in selected cell lines and restored Bmi1 mediated miR-200c expression inhibition. Recent study showed Bmi1 could lead to p53 protein downregulation via interaction mediated degradation [42]. Here, the inverse expression pattern of Bmi1 and wild-type p53 protein also was showed and coimmunoprecipitation assay showed the physical interaction, confirming the relationship. However, Bmi1 knockdwon also restored miR-200c expression in MDA-MB-231 and MDA-MB-453 cell lines with mutational p53, suggesting some other mechanisms responsible for Bmi1 mediating miR-200c regulation context dependently, which will be explored in our further study. As for expression regulation of miR-203, Zhang [43] et al have found the promoter hypermethylation responsible for miR-203 downregulation in metastatic breast cancer cell lines. However, whether promoter methylation is involved in miR-203 expression regulation in acquired anti-cancer drug –resistant breast cancer cells requires further inverstigation. Furthermore, the details on how Bmi1 regualted BCSCs mediate chemotherapy response also require further exploration.

Collectively, here we showed the important role of Bmi1 in breast cancer drug resistance and Bmi1-miRNAs cross-talk partially maintained the high expression of Bmi1. The present data implies new potential strategy with Bmi1 interference to promote the effect of chemotherapy for breast cancer.
